# Teachers’ perspectives of utilizing distance learning to support 21st century skill attainment for K-3 elementary students during the COVID-19 pandemic era

**DOI:** 10.1016/j.heliyon.2023.e19275

**Published:** 2023-08-24

**Authors:** Halah Ahmed Alismail

**Affiliations:** Faculty of Education, Curriculum and Instruction Department, King Faisal University, Al Ahsa 31982, Saudi Arabia

**Keywords:** Distance learning, Elementary school students, 21st century skills, Challenges, COVID-19

## Abstract

During the COVID-19 pandemic, Saudi Arabia, similar to other governments, discontinued face-to-face learning in favor of distance learning. The pandemic has had serious ramifications for K-3 education, and the impact of distance learning on 21st century skill attainment are important issues to explore. Using the Saudi Arabia context, this paper investigates teachers’ perspectives regarding the implementation of online education to support 21st century skills in the COVID-19 pandemic era for K-3 elementary school students. A qualitative research methodology was applied in this study. A semi-structured interview was conducted to collect data from five K-3 female teachers who implemented online education during the pandemic. Three themes emerged from the findings: 1) effects of the pandemic as related to online teaching for attainment of 21st century skills, 2) elaboration of best practices for online teaching to facilitate such attainment, and 3) challenges that exist for distance learning and student acquisition of 21st century skills. Therefore, the findings suggest that elementary teachers should find opportunities for elementary students to experience distance learning as an ongoing learning solution in order to incorporate innovative strategies that enhance their 21st century skills.

## 1 Introduction

The coronavirus disease 2019 (COVID-19) is an infectious disease caused by the SARS-CoV-2 virus [[1], [2], [3]], which first appeared in China in 2019 and rapidly spread worldwide, creating a health crisis that was soon labeled a global pandemic. Measures were implemented globally to limit the spread, which resulted in all public schools closing. The educational implications of this step were immense. By April 2020, 90% of the global student population was engaged in distance learning, with 192 countries completely closing all educational organizations [4]. Schools are now open, given the availability of COVID-19 vaccinations, and have resumed regular operations. However, the impact of COVID-19 on society has lasting and serious ramifications. Student learning during the COVID-19 pandemic required a rapid shift from classroom learning to distance learning due in part to social distancing policies to prevent the transmission of COVID-19 [[5], [6], [7]]. The need for social distancing advanced a rapid redesign of educational processes for which digital resources were prioritized [8]. The current paper addresses the need to better understand elementary teachers’ perspectives regarding how K-3 students can acquire 21st century skills within the COVID-19 distance learning context, particularly students under the age of 12 enrolled in the public education system [9].

When considering the special problems, issues, and obstacles that are unique to this age group, the emphasis on K–3 settings during the COVID-19 epidemic becomes more important [10]. Young kids need early skill development in 21st-century abilities to prepare them for the future, as the world is evolving quickly [9]. Recent studies have emphasized the value of cultivating not only the fundamentals of literacy and numeracy but also abilities like teamwork, critical thinking, problem solving, and digital literacy [11,12]. Age-appropriate pedagogical strategies that encourage the development of these skills must be given priority in distance learning. Young learners have shown potential for becoming engaged and developing 21st-century abilities using interactive and project-based learning techniques that incorporate digital tools and resources [13].

Additionally, parental support is essential in facilitating K–3 kids' distant learning opportunities throughout the pandemic. It is crucial to treat parents as partners in the education of their children and to give them the information and tools they need to get involved. In remote learning situations, parental participation has been shown to improve academic performance, motivation, and wellbeing [14,15]. Parental involvement can be increased and a supportive home learning environment can be created through collaborative efforts between teachers and parents, such as regular contact, parent workshops, and easily available learning resources [16].

Additionally, the COVID-19 epidemic has made already difficult problems worse, such as the digital divide, which limits everyone's access to online learning possibilities. To solve this problem, efforts should be undertaken to give all K–3 pupils equal access to technology and internet connectivity. Initiatives that give equipment, internet connections, and technical help to students from underprivileged backgrounds are important, according to recent studies [[16], [17], [18]]. To accommodate various learning demands and maintain inclusivity, educators might also think about alternative content delivery strategies, including offline resources and low-tech solutions. Given the COVID-19 pandemic's concentration on K–3 environments, it is critical to address the special issues and difficulties that are relevant to this age range. This entails highlighting the value of early 21st-century skill development, using age-appropriate educational strategies, and encouraging parental engagement [19]. By taking these factors into account, educators and decision-makers may develop a friendly and welcoming distance learning environment that gives young students the skills they need to succeed in a changing global context. The remainder of the Introduction details teachers' beliefs regarding the impact of COVID-19 on students' acquisition of 21st century skills and how this has impacted the education of K-3 elementary school students in Saudi Arabia. The following research questions are explored.

1. How have K-3 teachers supported 21st century skill acquisition during the pandemic within the distance learning context?
2. How do teachers experience the effectiveness of distance education during the COVID-19 pandemic on 21st century skill acquisition for K-3 students?
3. What distance learning challenges exist for teachers, and do these challenges impact the acquisition of 21st century skills in the context of the pandemic?

## 2 Literature review

### 2.1 21st century skills in elementary school

Skills students should learn in school in order to prepare to work and live in their society are referred to here as 21st century skills and require integration of essential training across the entire curriculum. Erdoğan [20] described 21st century skills as important for success in college, professional development, and social and professional life outside of academia. Additionally, the digital learning system has been proposed as an alternative technology-based learning solution that can be accessed by teachers and students using an online learning system [21]. These skills must be taught from elementary to secondary school using distance-based learning applications [22]. Consideration of 21st century skills in primary education is particularly important, given the rapidly changing conditions of one's personal, social, and professional life. Skills for the future were first recommended by John Dewey, who proposed an education “grounded in experience” in which students interact with the “ever changing world” [23]. A true visionary [24], defined an educated person as “one who thinks and reflects before acting, responds intelligently to a problematic situation and finally assesses the consequences of a chosen plan of action”. Clearly, this definition also describes a 21st century learner. Educators should foster communication and collaboration skills and think through how technology can be used. These innovations are important for students to learn how to critically think and solve problems. As such, 21st century skills should be integrated throughout the entire curriculum.

According to the Common Core State Standards Initiative [25], 21st century skills are 12 abilities, which align and support Bloom's taxonomy that students need to acquire in order to succeed in their future careers. Importantly, when teachers apply strategies that align with Bloom's taxonomy, they support students' capacities in critical thinking, independent learning, cooperation, and social interaction [26]. These skills are critical thinking, creativity, communication, collaboration, information literacy, technology literacy and media literacy, leadership and flexibility, initiative, productivity, and social skills. According to Fadel [27], 21st century skills are categorized as follows: a) learning and initiative skills, b) digital literacy skills, and c) life and career skills. These skills can help students keep up with new demands in the career markets but are dependent on the internet. The Partnership for 21st Century Skills a leading advocacy organization—works to promote the integration of 21st century skills in a larger educational framework that describes the skills and knowledge students need to acquire to contribute meaningfully to the workforce. Components of this framework are briefly described below.

First, *learning and initiative skills* includes four subskills: critical thinking and problem solving, innovation and creativity, communication, and collaboration. Critical thinking and problem solving can lead to creativity and innovation, and Bloom's taxonomy includes innovative thinking.

According to Luxton-Reily et al.'s literature analysis [28], Bloom's taxonomy is frequently used as a standard for evaluating students' learning in basic programming research. The researchers discovered that constructivist learning theories, theories of knowledge acquisition, and theories of self-regulated learning were all applied to students' transition from exploration to computational thinking [29]. The framework being offered highlights the importance of the cognitive load theory, which contends that learning falls with time when students are asked to remember an increasing number of things that are beyond the scope of their working memory.

As such, educators should allow students to apply, analyze, synthesize, and evaluate new information. As recommended by Partnership for 21st Century Skills [30], educators can provide opportunities for students to discuss and analyze different real-life topics and issues, allowing students to investigate problems, provide explanations, generate ideas, analyze data, and make judgments to solve a problem, thereby enhancing critical thinking skills [23,26,31]. Regarding the collaboration subskill, students work together to achieve a common goal, target the same objectives, and use communication skills to disseminate their ideas and innovations widely through various communication channels [32,33].

The second component *digital literacy skills* recognizes the need for a workforce experienced with digital technologies, and the ability to apply digital technologies to research, organize, evaluate, and communicate information to larger audiences [34]. The component comprises three literacy-focused subskills: technology, information, and media. Information literacy provides students with tools that allow them to distinguish between fact and fiction. Media literacy involves analyzing media and understanding problems that may arise while using the digital tools [35]. Technology literacy is obtained when students understand various applications and know when to use which methods and techniques and how to use them [32,33]. Torun [36] proposed that as digital technologies become more widely integrated, the educator needs to intentionally guide students within digital-rich classrooms that provide increasingly complex and diverse learning opportunities compared to the traditional classroom. Technological tools offer students the option of working in collaborative groups, which may support student motivation and increase critical thinking [36,37] and provide opportunities to expand their knowledge and experience through various means to understand the real world. This approach can help teachers enhance current lessons and facilitate discussion about the topics presented by using technological tools, making abstract or conceptual content more understandable [38]. Educators can be supported in advancing these skills through professional development, skills-specific training, and the allotment of time for designing technology-based lessons [39].

The third component of the framework *life career skills* includes comprises five subskills: flexibility and adaptability, leadership and responsibility, initiative and self-direction, productivity and accountability, and social and cross-cultural skills [40]. Flexibility and adaptability involve skills required to adapt to change and integrate complex views that impact decisions. Leadership and responsibility encompass an individual's ability to guide and influence others to achieve a goal. Initiative and self-direction guide students toward project initiation, project management and production, and the execution of strategies. Productivity and accountability assess an individual's potential to engage in their world and manage their work successfully across time [41]. Social and cross-cultural skills relate to students' abilities to encourage and motivate interaction with other people, particularly large groups of diverse people from various social backgrounds [27,40]. This framework recognizes that students in both online and offline environments should be experienced in communicating and collaborating with others. As technology skills become increasingly important, students benefit from activities that invite online discussions and internet use to learn and discuss with their peers. Offline communication opportunities are fostered as students become more collaborative and solve problems, engage in inquiry-based activities (such as science experiments), or research a particular topic [42]. In these contexts, group work is more creative, as it involves the integration of students' strengths and talents to accomplish a shared goal and every person in the team contributes [29]. Trilling and Fadel [43] emphasized that group work advances important social skills, such as mutual respect, timeline planning, and efforts toward compromising among team members. This form of cooperative learning advances student motivation [44] and peer-to-peer learning [43].

### 2.2 Saudi Arabia's COVID-19 response and educational implications

Following suit with other countries, Saudi Arabia physically closed all public schools in response to COVID-19 and utilized virtual and online learning and instructional practices as alternative approaches to in-person education strategies and activities [45]. Led by the national government, with particularly strong engagement from school administrators and educators, Saudi Arabia implemented full-time distance learning for all students for nearly a year from March 8, 2020 to August 29, 2021 [46]. In 2020, Saudi Arabia launched the Madrasati platform, which accelerated the time students were required to learn the distance learning platform system [1]. The Madrasati platform provides students and teachers a varied suite of applications for, among other things, conducting lessons using video conferencing, creating and completing assignments and quizzes, and generating reports. At the same time, Saudi Arabia launched the Ein platform. Supported by the Ministry of Education, this platform serves students, parents, and educational cohorts. A third platform the Ein Al-Mubdaa platform or the Creative EYE works to provide distance learning training courses and consultations [39]. Saudi Arabia's success in quickly implementing e-learning for students has been suggested to be due to the coinciding digital transformation in the country [1].

### 2.3 Saudi Arabia's implementation of distance learning

Distance learning has been conceptualized as multifaceted and covering many applications [47]. Utilizing the internet in online learning is paramount to successful implementation of distance learning and can provide students access to the materials provided and meetings [48,49]. Adam et al. [3] defined distance learning as any learning enabled electronically. Al-Khayyat [50] proposed that distance learning is composed of two types of learning: e-learning and computer learning. Students can deliver, receive, and choose learning programs, given the flexibility of time and place [51]. A 2018 study found that Saudi Arabia was successfully prepared to implement distance learning [52]. An analysis of surveys of school principals (TALIS) and students (PISA) revealed that in Saudi Arabia, educators were more open to change than those in other parts of the world. As such, there are opportunities for collaboration and professional development by using technology. Saudi Arabia will learn from the impacts of the COVID-19 pandemic and update school policies to respond to emergencies more efficiently.

## 3 Theoretical framework

The main theoretical frameworks for this study are constructivism and collaborative online learning. In the constructivist online environment, students create their own knowledge based on their cultural experiences, current circumstances, and viewpoints. In online learning environments, cultural constructivism encourages teachers to recognize all students' cultural viewpoints and strengths. Students are encouraged to share, engage in, contribute to, and discuss content through online collaborative learning. For instance, Goodfellow and Lamy [53] noted that one difficulty with constructivist theory in online learning is that teachers might not be aware of the students' cultural backgrounds and the experiences they bring to the setting.

According to Refs. [54,55], one of the most important elements that might influence how students view collaboration, communication, and group behavior is culture in online collaborative learning. Students have the chance to develop and improve their understanding through collaborative learning when they participate in knowledge production in online discussions [56]. According to studies by Refs. [57,58], computer-supported collaborative learning (CSCL) gave students the chance to develop a new socially associated knowledge-building structure that would enable them to participate in the development of knowledge in the online learning environment. However [59], discovered that not all students meaningfully contribute to the process of knowledge construction.

Additionally, the evaluation is meant to serve as a guide and a point of reference for future instruction. The five aspects of distant learning were aligned with Marzano's new taxonomy of educational objectives, which was chosen as the theoretical foundation for distance learning evaluation [60]. Marzano claimed that the self-system, the metacognitive system, and the cognitive system along with the element of knowledge were the three basic systems that made up the human learning process. Marzano suggested a two-dimensional evaluation system in light of this. Knowledge made up the first component and was divided into three domains: information (facts, organizational ideas), mental procedures (intellectual skills, intellectual processes), and physical procedures (psychological skills, psychological processes). Knowledge was comprised of six types. Six of the three systems were included in the second dimension, which focused on process operation. The cognitive systems first through fourth functions were knowledge retrieval, comprehension, analysis, and utilization. The fifth function was the metacognitive system, and the sixth was the self-system [61]. In order to create the value judgment for the learning task, the self-system was used, the metacognitive system was adopted to create the problem-solving techniques and procedures, and the cognitive system's fundamental cognitive abilities were used to accomplish the task [62]. These three systems were dependent on the supporting foundation of the knowledge field to function and work together. The theoretical frameworks mentioned above were therefore used to frame and direct this study.

Therefore, this paper focused on how the COVID-19 pandemic has influenced and changed the way that K-3 elementary school students learn and teachers teach, specifically using distance learning applications from the perspective of elementary teachers. In particular, this paper investigates the teachers’ perspectives of the implementation of online education to support 21st century skills in Saudi Arabia, considering the COVID-19 pandemic. As described, the pandemic required substantial changes in education systems that affected the Saudi Arabian educational landscape. The pandemic forced the realization that social distancing created a need for the redesign of teaching processes toward approaches in which distance learning is the norm and the new reality according to the information society [63]. Given the magnitude of this significant challenge, digital resources that can be proven to show better results than traditional teaching are necessary to support their implementation [8,64]. Similarly, the United Nations Educational, Scientific and Cultural Organization [65] has highlighted the need to promote quality education that adopts distance learning tools to be sustainable in education systems. With the need to rapidly pivot due to the pandemic, the priority of educational systems has been adoption of distance learning and e-learning and computer resources as a way to teach online [8]. Technology has already significantly accelerated educational systems and processes, and the pandemic will continue to accelerate the need for computer-based and distance learning processes [4]. As such, there is specific interest in perceptions about the potential of the online classroom to lead to the development of 21st century skills for K-3 elementary school students.

## 4 Methodology

### 4.1 Research model

A qualitative methodology was used in this phenomenological study to capture and explore the influence of the pandemic on teaching elementary students 21st century skills. The phenomenological method was selected to allow for an in-depth understanding of teachers’ perspectives [23,66]. The study was reviewed by the Institutional Review Board at King Faisal University, and ethical consent was obtained. All data were collected during the second semester between July 2021 and February 2022 in Saudi Arabia.

### 4.2 Participants

The approach for recruiting participants was purposive sampling, which is based on the assumption that the investigator will discover, understand, and gain insight. Vagle [66] recommended purposive sampling as an ideal selection method within phenomenological research. In this study, five female K-3 elementary teachers who used a digital platform to teach during the pandemic were selected. For the purpose of this investigation, which focuses on using distance learning to improve 21st-century skill achievement for K–3 elementary kids during the COVID-19 epidemic, only five female instructors were chosen. This decision was based on a number of important factors. First off, concentrating on female educators enables an exploration of their distinctive experiences, difficulties, and methods for adjusting to the requirements of distance learning during the pandemic. The study attempts to provide insight on the gender-specific dynamics that may affect teaching and learning in this context by looking at the viewpoints of female educators. Second, it discusses the significance of equity and representation in education. Studying female teachers' experiences helps give voice to their contributions and advance gender equity in the field because female teachers frequently encounter particular obstacles or underrepresentation. Additionally, using a smaller sample size of only five participants allows for in-depth data collection and analysis, enabling researchers to compile insightful data and explore the intricacies of the teachers' experiences. Although the sample size may restrict generalizability, it enables a thorough analysis of the strategies used by the chosen teachers to assist the development of 21st-century skills in K–3 students via distant learning during the COVID-19 epidemic.

Descriptive data of demographic characteristics, including grade level, gender, length of teaching experience, level of education of the teachers, and comfort with technology, are presented in Table 1.

**Table 1:** Profile of participants.

Variable	Frequency (%)
Nationality	
**Saudi Arabian**	5 (100%)
**Other**	0
Gender	
**Female**	5 (100%)
**Male**	0
Grade Level	
**Kindergarten**	1 (20%)
**1st**	1 (20%)
**2nd**	2 (40%)
**3rd**	1 (20%)
Years Teaching	
**1**–**5 years**	2 (40%)
**6**–**10 years**	1 (20%)
**11**–**15 years**	2 (40%)
Teacher Education Level	
**Bachelor Degree**	4 (80%)
**Master Degree**	1 (20%)
Comfort with Technology	
**Comfortable**	4 (80%
**Not Comfortable**	1 (20%)

### 4.3 Data collection and analysis

This study involved in-depth semi-structured interviews and field notes of the interviews. Notes were taken while listening, and the interviews were recorded and transcribed to confirm the notes taken [66,67]. In order to get further information about student success in this online course, semi-structured interviews were also conducted. The eight-question interview form was created around the major themes of the questionnaires used in this study. Two specialists in the fields of instructional technology at the schools looked over the interview questions. The teachers were asked to describe how they used technology before the COVID-19 pandemic and their current concerns (interview questions listed in Appendix A). Other areas explored include attitudes toward online learning, teacher motivation in applying distance learning in the classroom, distance learning challenges, and students' response to distance learning. Data were analyzed differently based on the type. Inductive coding allowed for derived codes from the qualitative data. The data were then broken into smaller data sets [20,23] and analyzed for themes. The coding process had a high reliability, as the researcher applied the code–recode strategy and coded twice [20]. The final codes and themes illustrate the teachers’ experiences and their perspectives of the phenomenon described by each theme [23,68].

### 4.4 Validity and reliability

Multiple obstacles could have affected the validity and reliability of this qualitative research study. The trustworthiness of qualitative research, which includes ensuring the research's reliability, dependability, and transferability, is typically addressed in the qualitative phase of this study. According to Lincoln and Guba [69], reliability is a critical factor to consider when assessing qualitative research. A key element of ensuring trustworthiness is establishing the legitimacy of qualitative findings.

Lincoln and Guba [69] provide a number of methods for building credibility. Peer debriefing, member-checking, and method triangulation were all used in this study to strengthen the validity of the qualitative results. In this study, five female K–3 elementary teachers who actively used a digital platform for instruction during the pandemic were chosen using a purposive sampling technique. The selection criteria took into account their subject-matter competence, participation in academic research, and support in qualitative research for K–3 elementary teachers. The peer researcher provided input that was integrated into the qualitative findings after rigorously reviewing every part of the qualitative phase of the study.

The researcher met in person with each of the five female K–3 elementary teachers who were being interviewed in order to ensure member checking during the qualitative phase. They were required to look at a thematic network diagram (see Fig. 1) that showed the main topics gleaned from the interviews. The goal was to determine whether the information shown in the network diagram truly reflected what the interviewees had said. Utilizing a methodological triangulation technique, the qualitative phase's credibility and dependability were increased. This involves using several techniques and data sources to validate the results and guarantee their consistency.

**Fig. 1:** Utilizing distance learning to support 21st century skill thematic analysis network.

## 5 Results

This study examined how K-3 teachers in Saudi Arabia experienced 21st century skill acquisition and curriculum delivery during the COVID-19 pandemic. To understand the scope of the phenomena, the participants were asked several questions during the interview process. During these in-depth interviews, the five teachers who agreed to participate shared their experiences with and perspectives regarding online education for 21st century skill attainment as related to their roles as educators. Review of the data obtained revealed three larger themes: 1) the effects of COVID-19 as related to online teaching for the acquisition of 21st century skills, 2) elaboration of best practices for online teaching to facilitate 21st century skills, and 3) Challenges that exist for distance learning and student acquisition of 21st century skills.

### 5.1 Theme 1: the effects of COVID-19 on online teaching for attainment of 21st century skills as realized through the pandemic response

The following interview question was asked: “How have teachers supported 21st century skill acquisition within the online learning context during the pandemic?” The interview process provided several insights into answering this question. Participants described different aspects of distance learning that had an impact on their students’ acquisition of 21st century skills. These perspectives can be described as four subthemes: 1) social distancing, 2) teacher–student relationship, 3) teacher motivation, and 4) student knowledge and capacity for using technology for education and 21st century skill attainment. These subthemes will be described below.

First is the requirement for social distancing. Teachers described how the widespread contagious nature of COVID-19 threatened the safety of teaching in person. However, the pandemic does not eliminate the need for teachers to deliver high-quality curriculum and learning for students to support 21st century skill acquisition. Important tools implemented in the virtual classroom included media, adapted methods, consideration of how to allocate and direct student at-home and independent study time, and how to ensure that learning strategies were properly implemented within online-learning system. The participants noted that the transitioning to a virtual environment limited their ability to read facial clues and the emotions of their students but increased 21st century skill acquisition. The participants reported that the pandemic, though limiting social interaction, has helped students become comfortable with distance learning and using technology. This is important for students as their future career paths and lives outside of school will likely involve technology and the ability to acquire skills in using technology. Therefore, distance learning provides an opportunity for all teachers. As one participant said

*After the pandemic, technology has become an integral tool in every level of education which gave students a chance to use technology and digital apps and being [*sic*] more confident with these digital tools often referred to as 21st century skills, especially life career, to be more able to be flexible and adapt to change and that we face during our lives.*

The participants expressed that as a learning medium, technology can facilitate active and student-focused learning. Though COVID-19 precautions forced schools to close, teachers were able to apply technology successfully through distance learning, which helped students become professionally oriented in digital skills, and use technology to communicate. Digital literacy skills became indispensable with face-to-face teaching phasing out because of the pandemic. As one participant described, the pandemic provided an opportunity for both teachers and students to be more comfortable with using technology and other digital tools and to become learners together in the digital space. Participants also reported that social distancing invited them to be innovative in how they teach. Flexibility and adaptability regarding curriculum and teaching methodologies were paramount to successful teaching, and tenants of leadership and responsibility guided motivation for both teachers and students. Additional facets, including initiative and self-direction, facilitate the execution of plans and are important aspects of the digital classroom. For example, one participant appreciated the flexibility distance learning allowed and the adaptability for handling unexpected conditions. Moreover, teachers found that distance learning helped their students be flexible in their relationships with their peers and that peer-to-peer learning was advanced. Important social skills, such as mutual respect, timeline planning, and efforts toward compromising among team members, were also advanced.

Within the second subtheme, the teacher–student relationship was deemed important. Participants discussed the significance of their relationship with their students and how they were motivated to use distance education to support students’ skills. Second-grade teachers talked about how they connected with their students during the time of COVID-19 and within the digital classroom:

*All of us had adapt to a new learning condition, which was distance learning. I encouraged my students to follow my lead as I directed them to communicate rules to address each other with respect virtually. Everyone is supporting each other, and our classroom became a family. Each of us participated, discussed, respected, and listened to the thoughts and ideas of others. From here, I work to improve students' skills and abilities, such as critical thinking, as well as develop creativity within my students.*

One participant mentioned that their relationship with students became better because of how they had to manage their classroom. The teacher worked to make the classroom friendly and positive, transforming it to a safe-space for truth-telling. They checked in often with their students to see how they were doing and what was going on in their lives, what they watched on TV, how their weekend went, and the types of things they said and did in an effort to increase motivation to think about how to encourage discussions and conversations. This participant noted,

*It was wonderful to experience with the students and have this unique experience. It can be a difficult time for many, but learning with the children was very important to learn how to be flexible and patient. I know it is important to organize my time and know that the topics up for discussion are numerous. There is nothing off table. All of this helps to create a very positive and happy relationship.*

Participants described their experiences developing and guiding student acquisition of 21st century skills while building a good relationship with their students. Participants said that they spent more time with their students. For example, one participant reported that their relationship with their students improved and that they used options such as emails, phone calls, and messages. For the participants, these kinds of relationships enhanced their effectiveness.

Teaching motivation was also identified as an important subtheme. The implementation of distance learning during the pandemic allowed for the experience of both ups and downs in teachers' motivations related to conditions that were brought on by the pandemic. Changes in the learning environment and the increase in the number of students and teachers affected by this pandemic both altered lifestyles and muted the enthusiasm to execute work-related activities. High motivation is crucial for teachers to have during online learning because the complexity of instruction through distance learning requires teachers to quickly overcome problems in virtual classrooms. One participant found that online learning encouraged teachers to be more creative and use different teaching strategies to help students to engage and focus. This increased students' motivation because they had the freedom and space to study on their own time and move around without restrictions or follow the classroom's role.

One participant expressed challenges with online learning due to the lack of in-person communication, which made it difficult to gauge how students were understanding the curriculum:

*I like teaching in person, learning, and meeting face to face because it allows me to interact directly with students and see them, which helped [*sic*] me also feel their joy. The relationship between my students was not as strong as before, and I struggled to maintain and build relationships with the ease that I experienced in the in-person classroom.*

Participants expressed that distance learning aided discussions of various topics related to both the pandemic and daily events and world news. These discussions led to new understandings about the COVID-19 vaccination, preventive measures, and how to best spend time while social distancing. This increased student motivation to learn, and students found that understanding and discussing the news increased their participation in class activities and enhanced their skills. Participants respected their peers and honored their independence and autonomy, as they had to wait for their turn to talk. Students showed more self-control and were more motivated to contain impulses and focus on the tasks at hand. Additionally, distance learning improved the teacher–learner–family relationship, which contributed to enhanced social skills and problem solving. One participant reported that learning through digital platforms increased their students’ self-direction and motivation because they had to use themselves as a resource and utilize resources they had at their disposal, such as smartphones, computers, tablets, and internet access. As one participant noted,

*As teachers, we work very hard to support students' learning and their motivation and learning performance; it helps to encourage a better education environment. All of this encourages students to be more responsible during [the] learning process and increase their abilities to learn in the virtual learning environment.*

Regarding the fourth subtheme student knowledge and capacity for using technology for education and 21st century skill attainment—the interview question posed was “How do you think the COVID-19 pandemic assisted in elevating the need and utility of learning 21st century skills through distance learning?” The participants discussed how in-person interactions were important and how online education increased students’ awareness of the importance of the online system as a significant alternative education option needed through the lockdown. Students learned to understand their roles and be innovative in obtaining the learning outcomes. The participants indicated that the cooperative learning model was beneficial. There are three main components to the cooperative learning model: a) improvement in student performance, b) opportunities for students with diverse backgrounds and abilities, and c) attainment of cooperation and collaboration skills.

### 5.2 Theme 2: elaboration of best practices for online teaching to facilitate 21st century skill acquisition

The second interview question that revealed evidence for the theme involving best practices was “How can distance learning support 21st century skills in K-3 elementary students?” All participants reported both negative and positive effects on social skills. The teachers noted that online education increased students' attention in learning and enhanced students' 21st century skills. Some positive impacts of the pandemic on distance learning included the opportunity for teachers to enhance and tailor training to match students' abilities. Participants applied technology for the acquisition of social and technical skills. One participant explained that distance learning helped connect lessons with real life by using pictures and videos downloaded before the COVID-19 pandemic. All participants agreed that instructional videos were one of the most effective media tools to apply in online learning because of available time and the ease of understanding the subject matter and how this was connected to the real world. Important here was that the instructional media related to the media students were exposed to at home and media that parents could utilize to connect with and improve the teacher–learner–family relationship. Together, this built the students’ literacy skills.

The participants confirmed they were responsible for designing projects and providing opportunities for discussion in their class design, supporting collaborative learning. The participants also cited negative effects of distance learning. For instance, there was not as much time to teach, which influenced the pace of learning, instructional objectives, and learning assessment. Time constraints and issues with internet access were also highlighted as factors for decreased efficiency. The use of online applications allowed only the most important points of a subject matter to be delivered to students. Also, how to approach late assignments and homework contributed to delays in instructional time. As one participant noted,

*I did not feel comfortable lecturing young students because they did not understand some concepts that needed to be learned face to face. Everything is limited, such as bad signals, quota availability, and students were not always prepared. In this way, their communications and interactions were not as good, and I could not tell if they were paying attention or not.*

### 5.3 Theme 3: challenges that exist for distance learning and student acquisition of 21st century skills

Additional challenges that participants faced are described here under three subthemes: technical obstacles, online teaching experience, and student conditioning. Within technical obstacles, challenges included the implementation of distance education, internet availability, and access to technology hardware. Not all parents owned the necessary technology, and some experienced poor internet signal, especially in the suburbs. Participants indicated that some students from low-income families could not provide laptops for their children, so students had to work from a smartphone or share a device with their siblings, which made distance learning a tedious process. As a result, some students experienced delays in completing assignments. Additionally, the lack of experience with using technology was often an issue. As one participant noted,

*Using distance education was difficult at first because I was used to in-person classrooms. It has become better, but I wish that I had more digital literacy before the COVID-19 pandemic began. Sometimes, I am challenged because I do not have the technology skills I need, and I cannot teach through [an] online [platform] because I have never taught virtually.*

Another challenge was student conditioning. Participants described barriers arising from the students' home environments, such as being distracted by family members. External factors had a significant impact. For example, disturbances from other students and family members when implementing learning using an online application, thereby becoming a crowded virtual environment, could become problematic. Participants also found it challenging to judge affective aspects of students' attitudes due to differences in attitudes between school environment and home learning. Participants explained that not being face to face impeded their ability to read their students’ emotions and that this contributed to reduced social skills. As one participant said,

*At the beginning of the pandemic, students were enthusiastic, but after two months, students were bored because they missed the physical interaction and communication with others. I was worried that if this continues, it will have a poor effect on social skills.*

These challenges impacted students’ learning and 21st century skill attainment. These challenges introduced technical barriers and obstacles that impacted online learning and posed a risk to the delivery of high-quality learning to condition students so they may be prepared to obtain important skills in the future.

## 6 Discussion

This study provided insights into online education during the pandemic and the impact of the pandemic on K-3 elementary school students' 21st century skill attainment in Saudi Arabia through their teachers’ perspectives. Several important impacts related to how 21st century skill attainment could have been facilitated in the distance learning context necessitated by the COVID-19 pandemic were revealed.

Distance learning significantly reduced in-person interactions between the students and teachers. As such, teachers were unable to observe their students’ emotions. Implementation of online classes contributed to reduced social contact, while the online learning system provided a means to ensure students could keep learning. Teachers within the distance learning context supported their students in being flexible and adaptable to change that was necessary due to the pandemic. Students experienced distance learning as a solution to ongoing learning using many different types of online platforms. Given the global nature of COVID-19, the need to shift to online education in the educational institutions allowed students to successfully achieve media and technology skills [40]. Consequently, this study found that students improved digital literacy skills needed for their future academic and professional careers [32]. Thus, the findings of the current study suggest that distance learning can help students become professionally oriented in digital skills, facilitate communication, and improve the ability to access information using technology. Educational changes due to COVID-19 impacted learning and allowed both teachers and students to have authentic experiences that motivated collaboration using the latest technologies [64].

The new online instructional methods for student learning during the pandemic was impacted by time, how the technology was applied, and psychological and social factors that significantly impacted the teacher–student relationship. Students were motivated to become attentive and focus on conversations with their teachers and peers, engage in the virtual classroom, and reach out to individual students and family members, which was an experience for most of them. Time spent with students helped improve their communication skills and provided the confidence students needed to be motivated to achieve learning objectives and engage in self-directed learning. Torun [36] emphasized that students’ readiness and academic achievement is derived from self-directed learning and motivation.

Additionally, the findings of the current study indicate that different online platforms enhance student agency, cooperation, and collaboration skills, which are important for improving the learning process and boosting student morale. Stauffer [40] explained that the support and encouragement students receive from peers helps to create bridge and reduce the gap between students and enhance learning readiness. Peer collaboration is also essential for successful online learning and affects the development of students’ 21st century skills [27].

The current study found that online learning had some negative effects, given time constraints that required teachers to adapt their instruction techniques and apply materials to the special features of the virtual classroom. The teachers agreed online learning limits social skills but helped them to be flexible and creative in preparing their online classes compared with traditional learning. This study suggests that teachers that are flexible and adaptable will help their students understand and connect to reality. When students can see the connections between what they are learning and real life, they are more likely to understand and apply meaning to events in their lives [70]. The use of instructional technology made it easier for young students to understand the subject matter by introducing a different type of learning experience, such as videos that have a real-life connection. Linkages between content and reality lets students engage in the learning environment effectively and promotes critical thinking, problem solving, and collaborative learning skills important for future academic and professional success [40,71].

This study also found that technology was important for improving the teacher–learner–family relationship. For example, instructional media used during the pandemic supported 21st century skill attainment while increasing family participation and activity in the child's learning, which enhanced the academic progress of the students. As Lemay and Doleck [72] explained, media applications, such as social media or media with social features, can help parents cope with the availability of materials at home. Bond [3] indicated that the assistance that parents provide during online learning promotes healthy relationships among all parties. Johnson et al. [31] noted that distance learning had a positive impact on communication skills among K-12 students during the COVID-19 pandemic because of the ability of students to interact with technology and learning platforms fully and knowledgeably.

The teachers experienced some challenges with online learning that were exacerbated by the COVID-19 pandemic. These obstacles are related to technical issues, teachers' online teaching experience, and student conditioning. Access to the necessary digital devices and the internet was a challenge and presented inequalities in the learning process. As such, there was a significant lack of inclusivity. Some students were unable to acquire the devices and digital resources necessary to participate in distance learning. This finding supports another study that indicated many students did not have an equal opportunity to access school curriculum material [52]. For the digital environment, students must have access to and possess the ability to use technology and the internet [7,63]. Because of differences in technology ability and access, some students did not obtain the learning materials, hardware, or software necessary for successful distance learning. As such, these students were disadvantaged, which had a negative impact on 21st century skill attainment [4]. Lastly, teachers indicated their lack of experience with technology as a challenge. Teachers’ use of technology and ability to implement distance learning indicates how smooth instructional activities will go, and teachers that have difficulty using technology will find it challenging to implement a successful digital classroom because of the requirement that teachers should master a great deal of online platforms. As such, it is important that teachers are trained and have technology skills, a realization that was made evident due to the COVID-19 pandemic [[73], [74], [75]]. This study also made the additional and surprising discovery that getting students to take part in online learning is difficult. Due to the distractions caused by family members and the home environment, children occasionally find it difficult to concentrate on the teacher. K–3 students were confused about what the educational setting should be after moving from a classroom to a home situation.

• Greater student collaboration: The study may show that online learning encourages more student collaboration among K–3 pupils than was previously thought. The design of virtual group activities and the development of cooperation abilities using online platforms and technologies may be affected by this unanticipated outcome.
• Improved creativity and problem-solving abilities: The study may show that the virtual learning environment fosters young students' capacity for original thought and the development of powerful problem-solving capabilities. This surprising result may encourage teachers to include more open-ended and inquiry-based exercises that develop these abilities in online learning environments.
• Improved student digital literacy: The study might uncover that K–3 pupils are more adept than predicted at using digital tools and resources. This unexpected outcome can serve as a reminder of the significance of including digital literacy as a foundational ability in early education and looking into strategies to improve kids' technological proficiency.
• Greater parental involvement and support: According to the research, K–3 pupils enrolled in distant learning must also have greater parental support. This surprising result can highlight how crucial it is to give parents access to tools, advice, and lines of contact to encourage their active participation in their child's virtual learning experience.

The consequences of these unexpected findings can help educators, curriculum designers, and policymakers evaluate and improve their methods for distance learning in K–3 environments. To provide successful support for students' distance learning experiences, it can encourage the inclusion of more cooperative and creative learning opportunities, the integration of digital literacy into the curriculum, and the development of better collaborations between schools and families. Overall, by making use of the study's findings, educators, administrators, policymakers, and parents may work together to improve distance learning procedures, address the problems found, and give young students valuable educational experiences even in remote locations.

## 7 Limitations and recommendations

This study has limitations, including the small representation of K-3 female teachers only who teach distance learning in Saudi Arabia. This limited how much could be discovered regarding the impact of this pandemic on 21st century skills in elementary school students. Thus, considering Vagle's [66] study, there is an inability to generalize findings with these participants' deep lived experiences. Future research could use different methodologies—including interviewing students and educators, along with parents and leaders of the Ministry of Education, on the implementation of virtual learning the pandemic. The research could be expanded to other provinces in Saudi Arabia. Finally, this study was confined to one geographical region. It is hard to say if the results can be generalized to other parts of the world.

## 8 Conclusion

This phenomenological study captured and explored online education in Saudi Arabia during the COVID-19 pandemic. The pandemic affected education and forced the redesign of teaching processes toward approaches in which distance learning is the norm and the new reality according to the information society [31]. With the need to rapidly pivot, distance learning became the standard teaching mode during the pandemic, beginning in February 2020. In Saudi Arabia, changes in the instructional system during the pandemic impacted how teachers taught and students learned, and technology readiness became vital. This study provided insights into distance education and the 21st century skills of K-3 students during the pandemic, as revealed through teacher interviews. The teachers indicated they could teach their students 21st century skills through distance learning strategies and tools. Because students were working from home, it became easier to teach new skills [47]. In this study, the teachers’ experiences demonstrate that distance learning platforms facilitate the development of specific skills, including innovation, collaboration, and communication skills, through indirect methods by using technology tools [7]. The digital environment reflects and allows many advanced technical skills and abilities. Concerted efforts of e-learning and computer transformation require innovation to ensure K-3 students can work as teams of scientists, mathematicians, designers, or other kinds of expert problem solvers.

## Author contribution statement

Halah Ahmed Alismail: Conceived and designed the experiments; Performed the experiments; Analyzed and interpreted the data; Contributed reagents, materials, analysis tools or data; Wrote the paper.

## Funding statement

The authors acknowledge the Deanship of Scientific Research, Vice Presidency for Graduate Studies and Scientific Research at King Faisal University, Saudi Arabia for financial support under the Annual Funding track [GRANT 3/924].

## Institutional Review Board statement

The study was conducted according to the guidelines of the Declaration of Helsinki, and approved by the Institutional Review Board (or Ethics Committee) of the Research Ethics Committee (REC) of King Faisal University (protocol code: KFU-REC–2022–DEC–ETHICS1,248).

## Data availability statement

Data included in article/supp. Material/referenced in article.

## Additional information

No additional information is available for this paper.

## Declaration of competing interest

The authors declare that they have no known competing financial interests or personal relationships that could have appeared to influence the work reported in this paper.

## Figures and Tables

**Table:** 

List of questions to individual teachers	
1.	What are 21st century skills that K-3 students should be learning?
2.	Why are these skills so important for young kids?
3.	How can distance learning support 21st century skills in K-3 Elementary students?
4.	How did COVID-19 change the way you teach 21st century skills?
5.	How did COVID-19 change how students learn and obtain 21st century skills?
6.	What do you believe about the distance learning and the using platform, was it good or bad?
7.	Do you think the students were preferred this way of teaching?
8.	From your experience, how do you use distance learning to support 21st century skills?
a) Can you provide an example?	
b) What is the challenge of distance learning for teaching and learning 21st century skills?	
c) What is the benefit of distance learning for obtaining 21st century skills?	
